The article "CDC20 May Serve as a Potential Biomarker-Based Risk Score System in Predicting the Prognosis of Patients with Hepatocellular Carcinoma" was retracted in 2023. Reasons: suspected computer-generated content; unreliable results or conclusions; concerns about the data; concerns about the results or conclusions.

# CDC20 May Serve as a Potential Biomarker-Based Risk Score System in Predicting the Prognosis of Patients with Hepatocellular Carcinoma

**DOI:** 10.1155/2022/8421813

**Published:** 2022-09-19

**Authors:** Qiliu Peng, Hai Huang, Chunling Zhu, Qingqing Hou, Shangmou Wei, Yi Xiao, Zhi Zhang, Xing Sun

**Affiliations:** ^1^Department of Clinical Laboratory, The Fifth Affiliated Hospital of Guangxi Medical University, Nanning, China; ^2^Department of Clinical Laboratory, Guangxi International Zhuang Medicine Hospital, Nanning, 530201 Guangxi, China; ^3^Department of Hepatobiliary Surgery, Guangxi Medical University Affiliated Wuming Hospital, Nanning 530199, China; ^4^Department of Spine Surgery, The Fifth Affiliated Hospital of Guangxi Medical University, Nanning, China; ^5^Departments of Hepatobiliary Surgery, The Fifth Affiliated Hospital of Guangxi Medical University, Nanning, China

## Abstract

**Background:**

The specificity and sensitivity of hepatocellular carcinoma (HCC) diagnostic markers are limited, hindering the early diagnosis and treatment of HCC patients. Therefore, improving prognostic biomarkers for patients with HCC is urgently needed.

**Methods:**

HCC-related datasets were downloaded from the public databases. Differentially expressed genes (DEGs) between HCC and adjacent nontumor liver tissues were then identified. Moreover, the intersection of DEGs in four datasets (GSE138178, GSE77509, GSE84006, and TCGA) was used in the functional enrichment, and module genes were obtained by a coexpression network. Cox and Kaplan-Meier analyses were used to identify overall survival- (OS-) related genes from module genes. Area under the curve (AUC) > 0.9 of OS-related genes was then carried out in order to perform the protein-protein interaction network. The feature genes were identified by least absolute shrinkage and selection operator (LASSO). Furthermore, the hub gene was identified through the univariate Cox model, after which the correlation analysis between the hub gene and pathways was explored. Finally, infiltration in immune cell types in HCC was analyzed.

**Results:**

A total of 2,227 upregulated genes and 1,501 downregulated DEGs were obtained in all four datasets, which were mainly found to be involved in the cell cycle and retinol metabolism. Accordingly, 998 OS-related genes were screened to construct the LASSO model. Finally, 8 feature genes (BUB1, CCNB1, CCNB2, CCNA2, AURKB, CDC20, OIP5, and TTK) were obtained. CDC20 was shown to serve as a poor prognostic gene in HCC and was mainly involved in the cell cycle. Moreover, a positive correlation was noted between the high degree of infiltration with Th2 and CDC20.

**Conclusion:**

High expression of CDC20 predicted poor survival, as potential target in the treatment for HCC.

## 1. Introduction

Hepatocellular carcinoma (HCC) is a familiar form and approximately 90% of all the liver cancers [1]. It is characterized by both phenotypic and molecular heterogeneity [2], and patients usually do not have significantly clinical symptoms during the early stages and are instead diagnosed when has developed to the middle and late stages. The diagnosis of HCC in the early stages has a relatively good prognosis and approximately accounted for 90% with a 5-year survival rate in surgery. If the diagnosis is made late, the postoperative survival rate is poor, and recurrence rate is high [3].

Biomarkers of miRNAs, genes, and lncRNAs have previously been reported in HCC patients. For example, highly expressed LHX3 is an independent prognostic factor of patients and serves as an advanced-stage prognostic biomarker in HCC [4]. miR-224 and miR-125b are also valuable prognostic biomarkers [5]. lncRNA-D16366 has been confirmed to be decreased in HCC [6]; nevertheless, lncRNA-D16366 in HCC diagnosis and prognosis remains unclear. These biomarkers may help in studying the prognosis of HCC while playing a complementary role in the clinicopathology of HCC [7, 8]. However, these biomarkers have not been researched in detail. Thus, clinical features closely related to the occurrence of HCC should be investigated to better predict prognosis while ascertaining potential prognostic markers.

The liver is an important organ in terms of immunity, where HCC cells can inhibit the immune system, leading to tumor cell proliferation and immunodeficiency [9, 10]. Furthermore, immune suppressor mechanisms favor tolerance over immunity and promote the progression of HCC [11, 12]. The immune microenvironment has been recognized to promote HCC metastasis and development [13], which has been shown to be correlated with poor prognosis in HCC. Therefore, in order to better understand the tumor-associated immune microenvironment, understanding the immune landscape of HCC is pertinent.

In this study, HCC tissues and adjacent nontumor tissues are used to analyze through a bioinformatics analysis from the public databases, including the Gene Expression Omnibus (GEO) database and The Cancer Genome Atlas (TCGA) database. The aim of this study is to screen the feature genes by LASSO along with the feature genes-based risk score to predict the prognosis of HCC with the hope of identifying potential targets in the treatment.

## 2. Materials and Methods

### 2.1. Data Preprocessing

RNA-sequencing raw data of 371 primary HCC and 50 normal tissues were obtained from the TCGA-Liver Hepatocellular Carcinoma (TCGA-LIHC) dataset (https://portal.gdc.cancer.gov/) [14]. Clinical information, including age, gender, grade, and overall survival (OS) of HCC patients, were collected. Public tumor microarray databases were obtained from GEO (http://www.ncbi.nlm.nih.gov/geo/) (accession numbers: GSE138178, GSE77509, and GSE84006) [15]. A total of 98 samples in the GSE138178, including 49 pairs of matched samples between HCC and adjacent nontumor liver tissues, were established using GPL21827 Agilent-079487 Arraystar Human mRNA microarray V4 (*Probe Name version*). The 98 samples obtained 70 male and 28 female, and the mean ages were 64.86 ± 11.21 [16]. A total of 60 samples in GSE77509, which consisted of HCC patients, each had three paired samples: primary tumor, adjacent normal tissues, and portal tumor thrombosis (PVTT). This study only focused on 20 primary tumor and 20 adjacent normal tissues, which were selected using GPL16791 Illumina HiSeq 2500 (*Homo sapiens*). The 40 samples obtained 34 male and 4 female, and the mean ages were 51.2 ± 8.41 [17]. A total of 152 samples in GSE84006, which consisted of 38 HCC tissues and 38 paired adjacent nontumor tissues, were established using GPL5175 Affymetrix Human Exon 1.0 ST Array [*transcript (gene) version*]. Among which, the 40 samples obtained 66 male and 10 female, and the mean ages were 52.87 ± 7.94. Meanwhile, the samples of GPL22109 were removed.

### 2.2. Screening of Differentially Expressed Genes

Abnormally expressed genes (in which expressed levels were too high or too low) were filtered to obtain expressed genes with at least 75% and a value of expression of more than 0 from TCGA. A differential expression analysis for gene expression between HCC tumor tissues and adjacent nontumor liver tissues in four datasets (TCGA, GSE138178, GSE77509, and GSE84006) was then performed using the limma R package [18]. Differentially expressed genes (DEGs) were identified out by setting the filter threshold adjusted *P* < 0.05 in all four datasets. The intersected DEGs of four datasets were identified by ggVennDiagram package [19] for the upregulated or downregulated DEGs. Finally, the cumulative distribution curve was drawn to identify the similarity of intersected DEGs in different samples from the four datasets.

### 2.3. Enrichment Analysis

To explore the biological processes and pathways involved in intersected DEGs, we constructed Gene Ontology (GO) terms and Kyoto Encyclopedia of Genes and Genomes (KEGG) enrichment analyses using clusterProfiler package [20] in R. *P* < 0.05 of the GO and KEGG were significant. A gene set enrichment analysis (GSEA) was then done in order to further explore the enrichment of intersected DEGs between HCC tissues and adjacent nontumor liver tissues. Moreover, the “fgsea” package in R displayed the results.

### 2.4. Construction of Coexpression Network

Weighted gene coexpression network analysis (WGCNA) could be a tool to identify the data, including looks for genes that have the same or similar expression patterns; structure of modules researches the relationships of modules and genes [21]. In this study, a coexpression network for intersected DEGs was used to construct by “WGCNA” package [21]. A sample cluster analysis was constructed using the “hclust” function, and modules were constructed using the “pickSoftThressholding” function, where the connectivity between the modules was evaluated (minModuleSize was 30). In order to further research the hub genes, a correlation analysis of the phenotype and modular gene was performed. The module eigengene could be the mean expression value of gene in a module. Genes with gene significance > 0.2 and module membership > 0.8 were known as hub genes in the module.

### 2.5. Analysis of Protein-Protein Interaction Network

Cox and Kaplan-Meier (K-M) curve analyses were used to confirm intersected DEGs in all four datasets that were closely associated with overall survival (OS) as OS-related genes in HCC. OS-related genes with *P* value < 0.05 are significant genes for further analysis. Next, area under the receiver-operating characteristic (ROC) curve of the module genes was identified in TCGA and GSE138178 using the pROC package [22]. Moreover, area under the curve (AUC) > 0.9 of module genes were used in order to establish the protein-protein interaction (PPI) network and were visualized using the Cytoscape software [23]. Molecular Complex Detection (MCODE) [24] was utilized to explore the vital modules in the PPI network with combined_score > 500.

### 2.6. Construction of Least Absolute Shrinkage and Selection Operator (LASSO) Model and Univariate Cox Regression Model

LASSO is a shrinkage model that can be used to reduce the likelihood of overfitting. The top 15 genes with a degree of significant module genes in the PPI network were used to construct the LASSO module with the glmnet package [25] in R, thus obtaining the most concise LASSO model. Specifically, 10-fold cross-validation was utilized to select the penalty term, in which *λ* calculates the binomial bias and serves as an indicator of the predictive capability of the model. Finally, the feature genes in HCC were obtained.

Univariate Cox regression analysis is mainly used to explore the independent prognostic effects of individual genes. Feature genes associated with prognostic genes were determined by the forestplot package in R. Here, feature genes with hazard ratio (HR) > 1 were considered significantly for prognosis.

### 2.7. Assessing the Ability to the Prognostic Risk Score of Feature Genes

The risk score of genes was used to assess the risk of individuals developing HCC. Here, the risk score was calculated for each patient and was predicted using the “coxph” function in the survival package [26]. Basing the median risk score, HCC patients were further divided into low/high-risk groups. Furthermore, a time-dependent ROC curve analysis was conducted at 1-, 3-, and 5-years in TCGA by the survival ROC package in R. Moreover, the rms package was used in order to construct nomograms, which are commonly used tools to estimate prognosis in oncology and medicine, and furthermore, calculated the consistency index and 95% confidence interval. Finally, the extent to which the predicted risk matches the actual risk was assessed using calibration curves.

### 2.8. Expression of Key Gene

The expressed key gene was explored as the study of external validation using Tumor Immune Estimation Resource (TIMER) (http://timer.cistrome.org/) databases, among which, the *P* < 0.001 and fold change > 1.5 as the selection.

### 2.9. The Level of Immune Cell Infiltrated in HCC

The infiltration levels of immune cells were highly related with both the progression and prognosis of HCC, in terms of tumor and adjacent nontumor tissues, to calculate immune cell infiltration using single sample Gene Set Enrichment Analysis (ssGSEA) by the marker gene sets [27]. Additionally, the correlation of immune cells was explored using the ggradar package and performing correlation analysis to further explore the significant correlation between the genes and immunity. To explore the differences of the immune cell types, we used the CIBERSORT algorithm (https://cibersort.stanford.edu/) to assess the proportion of 22 immune cell types [28] among the HCC samples.

### 2.10. Statistical Analysis

This study was involved in the analyses using the BioInforCloud platform (http://www.bioinforcloud.org.cn).

## 3. Results

A flow chart about the method of this study is shown in Figure 1.

### 3.1. Identifying the DEGs in HCC

Comparing nontumor tissues, 18101 DEGs were identified of HCC in GSE138178, including 9,923 upregulated and 8,178 downregulated genes (Figure 2(a)). A column diagram was made to visualize the counts of DEGs in the four HCC datasets (Figure 2(b)). The results showed the following among the datasets: 18,101 DEGs of GSE138178, 11,012 DEGs of GSE77509, 9,914 DEGs of GSE84006, and 12,675 DEGs of TCGA. Among them, there was a total of 3728 intersected DEGs in the four datasets, which consisted of 2,227 upregulated genes and 1,501 downregulated genes (Figure 2(c)). Gene expression similarity of the intersected DEGs were found to be the highest in the different samples in HCC of GSE138178 and GSE84006 (Figure 2(d)).

### 3.2. Biological Function of HCC

As shown in Figure 3(a), intersected DEGs were shown to be enriched in the cell cycle and AMPK signaling pathway. Biological process of intersected DEGs were found to be mainly enriched in DNA replication and ribosome biogenesis. Furthermore, the GSEA findings showed that intersected DEGs were mainly involved in the cell cycle, DNA replication, and mismatch repair, which was activated in HCC. Meanwhile, propanoate metabolism, retinol metabolism, and tryptophan metabolism were observed to be inhibited (Figures 3(c) and 3(d)). The activation of the pathways of intersected DEGs was enriched and that plays a role in promoting in HCC.

### 3.3. Module Genes Were Identified by WGCNA

Intersected DEGs were used to identify the module genes by WGCNA, which indicated that when the soft threshold power was 5, the independence was greater than 0.90 (Figure 4(a)). Nine coexpression modules were then obtained (Figure 4(b)), where the yellow module was found to have a significant positive correlation with HCC (Figure 4(c)). Furthermore, the hub genes in the yellow module were significantly associated with HCC (Figure 4(d)); the significant module genes were used for further analysis in subsequent studies.

### 3.4. Screening the Feature Genes Associated with Prognostic Genes

Intersected DEGs were used to identify OS-related genes in TCGA and GSE138178 by Cox and K-M curve analyses. The AUC values of OS-related genes in HCC of TCGA and GSE138178 are shown in Figure 5(a). AUC > 0.9 of OS-related genes were then used to perform the PPI network (Figure 5(b)). The 15 genes with the largest degree of connectivity in the genes of the PPI network were used to construct the LASSO model, after which 8 feature genes were identified (Figures 5(c) and 5(d)). All 8 feature genes (BUB1, CCNB1, CCNB2, CCNA2, AURKB, CDC20, OIP5, and TTK) were observed to have a poor prognosis in HCC, suggesting that the 8 feature genes could be a useful biomarkers of HCC prognosis (Figure 5(e)). Basing the LASSO model obtained 8 feature genes associated with prognosis, considering the feature genes play a vital role brings it to our attention in HCC.

### 3.5. Feature Genes as a Prognosis in HCC

A high- and low-risk group of HCC patients is basing the median risk score of the feature genes (Figure 6(a)). The 1-, 3-, and 5-year survivals of AUCs were found to be more than 0.65 (Figure 6(b)). Nomograms were used to quantify the risk factors of feature genes along with the 3- and 5-year survival probability. Interestingly, CDC20 was shown to have the worst prognosis, which indicated that CDC20 may be a hub gene for prognosis in HCC (Figure 6(c)). Furthermore, calibration plots were used to predict the ability of nomograms, which were shown to perform well (Figure 6(d)). Above all, we considered CDC20 has the worst prognosis, which may be a hub gene for prognosis in HCC.

### 3.6. Biological Process and Pathways of CDC20

The AUC for CDC20 was noted to be higher than 0.95 in all four datasets, which indicated that CDC20 has high diagnostic value for HCC (Figure S1A). Comparing the HCC and control samples in all four datasets, CDC20 was overexpressed in HCC (Figure S1B). Comparing the adjacent normal tissues, CDC20 was closely higher in HCC by TIMER database (Figure S1C). The enrichment analysis of BP showed that CDC20 had a positive correlation among the cell cycle, DNA replication initiation, and mitotic chromosome condensation, while fatty acid oxidation and megahydroxylase P450 pathway were negatively correlated in HCC (Figure 7(a)). Additionally, the KEGG pathways of CDC20 were found to be a positive correlation, which related with the cell cycle and DNA replication, but they were negatively correlated with the AMPK and PPAR signaling pathways (Figure 7(b)). CDC20 was also shown to serve as a downstream gene in the cell cycle (Figure 7(c)). In general, CDC20 has a positive correlation with cell cycle, which plays the part of positive regulation in HCC.

### 3.7. Hub Gene and Infiltration of Immune Cells

The levels of infiltration for immune cells in all four datasets were analyzed by ssGSEA, in which type-2 T helper (Th2) cells and T helper (Th) cells were found to have a significantly high degree of infiltration, while neutrophils, gammadelta T cells (Tgd), and cytotoxic cells had a significantly low degree of infiltration in HCC (Figures 8(a) and 8(b)). Moreover, a negative correlation of CDC20 and dendritic cells (DC) was observed through the correlation analysis (Figure 8(c)).  Figure 8(d) illustrates the positive correlation between CDC20 and Th2 cells. T cell CD4 memory resting was also identified to have the most degree of infiltration in all immune cell types in HCC (Figure 8(e)). The results indicated that Th2 cell, Th cell, and T cell CD4 memory resting has high degree of infiltration of HCC. Understanding the tumor immune microenvironment provides the basis of immunization therapy in HCC.

## 4. Discussion

Several studies have reported that certain prognostic genes may serve as predictors of OS for patients with HCC, such as a gene-based signature comprising of CDC6, CENPE, PIK3R1, KIF11, and RACGAP1 [29], which may be significantly associated to the poor prognosis of HCC. Nevertheless, these biomarkers are insufficient, and further exploration of biomarkers in HCC is necessary. In this study, a LASSO and univariate Cox model were constructed, where 8 feature genes were identified and associated with the OS. CDC20 was found to serve as the hub gene with a poorer prognosis according to the feature genes-based risk score. Furthermore, Th2 cells and DCs were shown to possess a high degree of infiltration by ssGSEA.

The intersection of DEGs were participated in the cell cycle and AMPK pathway. BP of intersection of DEGs were enriched in DNA replication and Fanconi anemia pathway in HCC. The previous studies indicated that AMPK pathway was downregulated to reduce the proliferation in lots of the cancer cells and obtained HeLa, prostate cancer cells [30, 31], suggesting that activation of AMPK signaling maybe promoted the progress for HCC. Various studies have reported that cell cycle arrest induction is done in order to attenuate tumor progression in HCC [32]. Additionally, interacted kinases may regulate DNA replication, repair, and cell cycle progression in HCC [33]. Notably, the expression of Fanconi anemia and double-stranded DNA break repair genes was found to be significantly upregulated in HCC [34]. These pathways may all play an important role in the development of HCC.

Meanwhile, the coexpression network analysis suggested that the yellow module was significantly correlated with HCC, and module genes may promote the development of HCC. As the prognosis of HCC is not optimistic, 998 OS-related genes were obtained via Cox and Kaplan-Meier curve analyses. Then, 152 OS-related genes of module genes with AUC > 0.9 performed the PPI network and LASSO model, in which 8 feature genes, including BUB1, CCNB1, CCNB2, CCNA2, AURKB, CDC20, OIP5, and TTK, were identified. These genes were then used to construct a univariate Cox regression module, where all feature genes were associated with HCC prognosis. Among them, BUB1, CCNB2, and CDC20 in tumor tissues were shown to have poor survival in HCC, which could be potential targets in the treatment for HCC [35]. BUB1, CCNB2, CCNA2, and TTK were found to be associated with HCC prognosis, which may serve as potential biomarkers of HCC [36]. Furthermore, a Cox regression model including OIP5 and AURKB may predict OS in HCC patients effectively [37]. Nomograms are widely used for cancer prognosis [38] in evaluating feature genes. Interestingly, among feature genes, CDC20 was found to have a poorer prognosis for HCC according to the nomograms. Moreover, the AUC value of CDC20 was found to be more than 0.95. In addition, compared with controls, overexpression of CDC20 was evident in the 4 datasets. Overall, CDC20 may serve as a biomarker for prognosis in HCC.

Approximately 40 years ago, CDC20 was primarily discovered to regulate cell cycle progression [39]. Recently, various researches have shown that CDC20 is overexpressed in different types of tumors. In comparison to normal cells, CDC20 is known to be overexpressed in breast cancer [40], cervical cancer [41], and glioblastomas [42]. In this study, a high expression and poor prognosis of CDC20 was noted in HCC, which was positively correlated with the cell cycle and DNA replication. Aberrant function of cell cycle regulators leads to cell proliferation, and some protein kinases of the cell cycle may also regulate DNA replication [43]. This suggests that protein kinase of the cell cycle may be involved in cell proliferation in the HCC cell cycle. Above all, CDC20 is a therapeutic target of drug development for the treatment of human malignancies [44].

HCC, as one of the most malignant liver disease, has a close relationship between environmental factors and tumor diseases [45] When comparing HCC and healthy samples, immune cell types were shown to be decreased in HCC samples. In contrast, immune infiltration levels of Th2 cells and Th cells were found to be strongly increased in HCC. The CIBERSORT algorithm calculated the proportions of immune cells, which showed T cell CD4 memory resting was the largest. Previous studies have shown that T cells, Th2 cells, NK cells, and macrophages are related with prognosis in patients with HCC [45]. Studies have also demonstrated that Th2 cytokine is involved in hepatitis C virus (HCV) pathogenesis and promotes the severity of liver disease [46]. Furthermore, a positive correlation was found to exist between Th2 cell and CDC20, which was noted to be related to OS in HCC. Accordingly, immunity with the cells and the microenvironment all could be the basal factors in the occurrence of tumors [47]. Therefore, CDC20 may act as a promising therapeutic target for HCC.

However, certain several limitations should be noted in this study. The data from public databases were used for bioinformatics analysis. Hence, additional studies are warranted to validate the clinical benefits of CDC20 in the treatment of HCC.

In general, the intersection of DEGs in the four datasets was constructed a coexpression network to screen 998 OS-related genes which were identified by Cox and Kaplan-Meier analyses. Perform the PPI network, and LASSO model screened 8 feature genes. Then, univariate Cox model and risk score demonstrated a high expression of CDC20 as a poor overall survival- (OS-) related gene in HCC patients. Furthermore, Th2 cell had high degree of infiltration with CD20 in HCC. Finally, we found that CDC20 was significantly correlated with the cell cycle in HCC. Therefore, we consider CDC20 as a vital marker in the prognosis in HCC.

## 5. Conclusion

Hub genes in HCC were identified through a bioinformatics analysis, in which overexpression of CDC20 in tumor tissues was shown to be predictive of poor survival and could be as potential targets in the treatment for HCC.

## Figures and Tables

**Figure 1:** Workflow of the study. In step 1, differentially expressed genes (DEGs) of TCGA, GSE138178, GSE84006, and GSE77509 between HCC and adjacent nontumor liver tissues were identified by differential expression analysis. Functional enrichment analyses were performed using the intersection of DEGs in the four datasets. In step 2, a coexpression network was done to screen the module genes, in which 998 OS-related genes were identified by Cox and Kaplan-Meier analyses using the module genes. An area under the curve (AUC) > 0.9 of OS-related genes was obtained by AUC analysis to construct the protein-protein interaction (PPI) network. In step 3, 8 feature genes were identified by least absolute shrinkage and the selection operator (LASSO) model. Then, univariate Cox model and feature gene-based risk score demonstrated a high expression of CDC20 as a poor overall survival- (OS-) related gene in HCC patients. In step 4, expression profiles of the four datasets were performed on the single sample GSEA to explore immune cell infiltration and the correlation of upregulated type-2 T helper cells and CDC20. In step 5, the correlation analysis of CDC20 and its biological pathways showed that the cell cycle was significantly correlated with CDC20 in HCC. AUC: area under the curve; DEG: differentially expressed genes; GSEA: gene set enrichment analysis; K-M: Kaplan-Meier; HCC: hepatocellular cancer; LASSO: least absolute shrinkage and selection operator; OS: overall survival; PPI: protein-protein interaction; ROC: receiver-operating characteristic curve; TCGA: The Cancer Genome Atlas. WGCNA: weighted gene coexpression network analysis.

**Figure 2:** Identifying the differentially expressed genes (DEGs) in HCC. (a) Identification of DEGs between controls and HCC samples in GSE138178. (b) DEGs of TCGA, GSE77509, GSE84006, and GSE138178 datasets. (c) Intersection of DEGs were upregulated and downregulated in HCC. (d) Cumulative distribution plots demonstrated the similarity of the expressed DEGs in four datasets. HCC: hepatocellular cancer; Log_2_FC; log_2_fold change. TCGA: The Cancer Genome Atlas.

**Figure 3:** Biological functions of HCC. (a) Intersected differentially expressed genes (DEGs) were involved in the Kyoto Encyclopedia of Genes and Genomes (KEGG) pathways. (b) Gene ontologies were mainly enriched by the intersected genes. (c) Intersected DEGs were predicted to activate in the top 6 pathways. (d) Intersected DEGs were predicted to inhibit in the top 6 pathways, as shown by GSEA. Defining the enriched genes as genes significantly expression of HCC tissues that indicated high enrichment scores. DEGs: differentially expressed genes; GSEA: gene set enrichment analysis; HCC: hepatocellular carcinoma.

**Figure 4:** Identification of module genes by WGCNA. (a) The scale-free network diagram of intersected DEGs. Left: distribution of network-free scales; right: mean of the gene adjacency function of the corresponding gene module. (b) Clustering dendrogram of intersected DEGs. Colors indicate different modules. (c) Heatmap shows groups of correlated genes termed modules. ME; module eigengene. (d) The module genes were observably correlated with yellow.

**Figure 5:** LASSO regression and univariate Cox models. (a) Predicting the AUC value of intersected DEGs. The 10 genes (red represents upregulated genes; blue represents downregulated genes) are shown with AUC > 0.95. (b) 152 module genes are shown by the protein-protein interaction network. (c) Coefficient of the 8 feature genes in regression model. (d) Crossing validation curve. (e) Univariate analysis of feature genes. AUC: area under the curve; HCC: hepatocellular carcinoma; LASSO: least absolute shrinkage and selection operator.

**Figure 6:** Exploring the prognostic biomarkers basing risk score. (a) HCC patients of the TCGA dataset were divided into different groups and A risk score, B survival status, and C expressed feature genes. (b) Time-dependent ROC of patients in the TCGA. (c) Nomogram for predicting survival for HCC patients with feature genes. (d) Calibration curves for feature genes and 3- and 5-year OS in the validation set (TCGA). HCC: hepatocellular cancer; OS: overall survival; ROC: receiver-operating characteristic curve; TCGA: The Cancer Genome Atlas.

**Figure 7:** Relationship of CDC20 and biological function. (a) Correlations of CDC20 and biological function. Red indicated the degree of activation, while green indicated the degree of inhibition. Sector indicated the correlation of CDC20 and biological processes. (b) Pertinency between CDC20 and pathways. Solid lines indicated positively correlated, while dotted lines indicated negatively correlated. (c) Role of CDC20 in the cell cycle.

**Figure 8:** The infiltration of the immune cell in hepatocellular cancer. (a) Levels of immune cell infiltration in the four datasets (TCGA, GSE138178, GSE84006, and GSE77509). (b) Radar plot shows the correlation of immune cell types in HCC. (c) Significantly negative correlation of CDC20 and dendritic cells. (d) Significantly positive correlation of CDC20 and type-2 T helper (Th2) cells. (e) Estimated proportions of 22 immune cell types.

## Data Availability

The dataset used and analysed during the current study are available from the corresponding author on reasonable request.

## Supplementary Materials

Supplementary Materials Supplementary Figure S1: the expression of CDC20 in HCC.
